The article "Impact of Dual Antiplatelet Therapy Versus Monotherapy in Acute Stroke Management: A Systematic Review" was retracted in 2025. Reasons: unreliable results or conclusions; concerns about the authorship.

# Impact of Dual Antiplatelet Therapy Versus Monotherapy in Acute Stroke Management: A Systematic Review

**DOI:** 10.7759/cureus.78138

**Published:** 2025-01-28

**Authors:** Muhammad Adil Areeb, Rakesh Mohanty, Hiren B Hisoriya, Javeria Mithani, Oluwatobiloba T Ogungbemi, Kesha Pathak, Umar Farooq, Rauda Al Dhaheri, Ahmad Zubair Aziz, Nishath Kausar, Ali Raza

**Affiliations:** 1 Neurology, Avicenna Tajik State Medical University, Dushanbe, TJK; 2 Anesthesiology, King's College Hospital, London, GBR; 3 Internal Medicine, Poona Hospital and Research Centre, Pune, IND; 4 Internal Medicine, Karachi Medical and Dental College, Karachi, PAK; 5 Internal Medicine, Caucasus's International University, Tbilisi, GEO; 6 Internal Medicine, Gujarat Adani Institute of Medical Sciences, Bhuj, IND; 7 Medicine and Surgery, Avicenna Medical College, Lahore, PAK; 8 Cardiology, Dubai Medical College for Girls, Dubai, ARE; 9 Internal Medicine, Hunan Normal University, Khanpur, PAK; 10 Internal Medicine, Sitara Medical Center, Hyderabad, IND; 11 Internal Medicine, Nishtar Medical University, Multan, PAK

**Keywords:** aspirin, cilostazol, clopidogrel, dual antiplatelet therapy, genetic polymorphisms, ischemic stroke, personalized medicine, stroke management, stroke recurrence, transient ischemic attack

## Abstract

This systematic review evaluates the comparative efficacy and safety of dual antiplatelet therapy (DAPT) versus monotherapy in the management of acute ischemic stroke and transient ischemic attack (TIA). Six studies, published between 2019 and 2024, were included, focusing on patient outcomes such as stroke recurrence, functional recovery, and safety measures. The findings consistently demonstrated that DAPT, particularly combinations like aspirin with clopidogrel or cilostazol, significantly reduced stroke recurrence and improved functional outcomes as compared to monotherapy, without a notable increase in major bleeding risk. Timing and duration of therapy were identified as critical factors, with early initiation and prolonged DAPT showing promising results in high-risk populations, including those with intracranial arterial stenosis or large artery atherosclerosis. Genetic polymorphisms, such as CYP2B6 variants, further influenced treatment efficacy, highlighting the potential for personalized therapeutic approaches. While the evidence underscores the clinical value of DAPT, it also identifies gaps such as the need for real-world studies and investigations into long-term safety. This review contributes to advancing stroke management by providing a nuanced, evidence-based perspective on the role of DAPT in reducing vascular events and disability.

## Introduction and background

Stroke is a leading cause of mortality and long-term disability worldwide, with ischemic stroke accounting for approximately 87% of all stroke cases [1]. Effective secondary prevention strategies are essential to minimize the risk of recurrence and to improve functional outcomes. Antiplatelet therapy plays a pivotal role in the management of ischemic stroke, as it prevents the aggregation of platelets, thereby reducing the risk of thromboembolic events [2].

The article "Impact of Dual Antiplatelet Therapy Versus Monotherapy in Acute Stroke Management: A Systematic Review" was retracted in 2025. Reasons: unreliable results or conclusions; concerns about the authorship.

Dual antiplatelet therapy (DAPT), which combines two antiplatelet agents, has been explored extensively for its potential benefits in reducing recurrent stroke compared to monotherapy [3]. However, the increased bleeding risk associated with DAPT remains a concern, necessitating a nuanced understanding of its benefits and limitations. Studies have evaluated different combinations of antiplatelet agents, such as aspirin and clopidogrel or cilostazol, in diverse patient populations to optimize therapy for acute ischemic stroke and transient ischemic attack (TIA) [4].

Recent evidence highlights the role of genetic polymorphisms, timing of therapy initiation, and specific patient subgroups (e.g., those with intracranial arterial stenosis or carotid disease) in influencing the efficacy and safety of antiplatelet strategies [5]. Despite advancements, there is ongoing debate regarding the optimal antiplatelet approach for acute stroke management. While several trials have demonstrated the potential benefits of DAPT, particularly for short durations, variations in trial outcomes and patient-specific factors contribute to the lack of consensus on its superiority over monotherapy. This systematic review aims to synthesize and critically evaluate the available evidence to address this knowledge gap, focusing on the impact of DAPT versus monotherapy on stroke recurrence, functional outcomes, and safety profiles.

The PICO framework (Population, Intervention, Comparison, and Outcome) was employed to formulate the research question and guide the selection of studies included in this systematic review [6]. The population of interest consists of patients with acute ischemic stroke or transient ischemic attack, with specific subgroups, such as those with intracranial arterial stenosis or nonstenotic carotid disease, considered to explore the differential impacts of therapies. The intervention examined is DAPT, including combinations such as aspirin with clopidogrel or cilostazol. This is compared against monotherapy using a single antiplatelet agent such as aspirin or clopidogrel. The primary outcomes of interest include stroke recurrence and functional improvements, such as reductions in disability, while secondary outcomes focus on the safety profile of these interventions, particularly the incidence of bleeding complications. This structured framework ensures a comprehensive and focused approach to addressing the key aspects of antiplatelet therapy in acute stroke management.

The article "Impact of Dual Antiplatelet Therapy Versus Monotherapy in Acute Stroke Management: A Systematic Review" was retracted in 2025. Reasons: unreliable results or conclusions; concerns about the authorship.

## Review

Materials and methods

Search Strategy

The search strategy for this systematic review was designed in accordance with the PRISMA (Preferred Reporting Items for Systematic Reviews and Meta-Analyses) guidelines to ensure a comprehensive and transparent selection process [7]. We conducted a systematic search across major electronic databases, including PubMed, MEDLINE, and EMBASE, to identify studies published within the last five years (2019-2024) in the English language. The search terms included combinations of keywords such as “dual antiplatelet therapy,” “monotherapy,” “stroke,” “ischemic stroke,” “TIA,” “clopidogrel,” “aspirin,” and “cilostazol.” Boolean operators (AND, OR) were employed to refine the search, and filters were applied to include only peer-reviewed articles. Additional manual screening of references from included studies was performed to ensure all relevant articles were captured. The screening process involved a title and abstract review, followed by a full-text evaluation to assess eligibility based on predefined inclusion and exclusion criteria. The systematic approach ensured a robust selection of high-quality studies directly addressing the research question.

Eligibility Criteria

The eligibility criteria [8] for this systematic review were established to ensure the inclusion of studies that directly addressed the research question regarding the impact of DAPT versus monotherapy in acute stroke management. Studies were included if they met the following criteria: (1) randomized controlled trials (RCTs) or post hoc analyses of RCTs examining the effects of DAPT, such as aspirin combined with clopidogrel or cilostazol, compared to monotherapy in patients with acute ischemic stroke or transient ischemic attack (TIA); (2) published in English between 2019 and 2024 to ensure recent and relevant findings; and (3) reported key clinical outcomes, including stroke recurrence, functional outcomes (e.g., modified Rankin Scale), and safety measures such as bleeding complications.

Exclusion criteria were applied to filter out studies that did not meet the focus of this review. Studies were excluded if they (1) were observational, retrospective, or not peer-reviewed; (2) did not provide sufficient statistical data on the efficacy or safety of DAPT versus monotherapy; or (3) included patient populations with stroke subtypes or conditions unrelated to the scope of the review such as cardioembolic stroke. Additionally, systematic reviews, meta-analyses, editorials, and commentaries were excluded to avoid redundancy and focus solely on primary research. The decision to exclude observational studies was guided by the aims of the review, which sought to synthesize high-quality evidence from RCTs to ensure reliability and minimize bias. While observational studies can provide valuable real-world insights, they are often subject to confounding factors and selection bias, which may affect the validity of the findings. These criteria ensured that only high-quality, directly relevant studies were included to provide robust and reliable insights for the review.

The article "Impact of Dual Antiplatelet Therapy Versus Monotherapy in Acute Stroke Management: A Systematic Review" was retracted in 2025. Reasons: unreliable results or conclusions; concerns about the authorship.

Data Extraction

Data extraction for this systematic review was conducted systematically and in alignment with PRISMA guidelines to ensure accuracy and reproducibility. A standardized data extraction form was developed to collect key information from each included study. Extracted data included study characteristics (author, year, study design, and population), intervention details (type, duration, and timing of DAPT), comparator details (monotherapy regimen), and outcomes measured (stroke recurrence, functional outcomes, and safety, such as bleeding events). Additionally, statistical data, including hazard ratios, confidence intervals, and p-values, were meticulously recorded to facilitate comparisons across studies. Two independent reviewers performed data extraction, with discrepancies resolved through discussion or consultation with a third reviewer to ensure consistency and minimize bias. The extracted data were synthesized to provide a comprehensive evaluation of the efficacy and safety of DAPT versus monotherapy in acute stroke management.

Data Analysis and Synthesis

The data analysis and synthesis process for this systematic review adhered to a narrative synthesis approach, guided by PRISMA recommendations, to ensure a structured and comprehensive evaluation of the included studies. Extracted data were analyzed qualitatively to compare the efficacy and safety of DAPT versus monotherapy across various clinical outcomes, including stroke recurrence, functional recovery, and bleeding risks. Quantitative data, such as hazard ratios and confidence intervals, were tabulated to highlight patterns and differences in treatment effects. Subgroup analyses were performed to explore variations in outcomes based on factors such as timing of treatment initiation, stroke subtype, and patient characteristics. The findings were synthesized to identify consistent trends, gaps, and areas requiring further research, providing a clear and cohesive summary of the current evidence on the impact of DAPT in acute stroke management. Statistical data were interpreted in the context of clinical relevance to inform practical recommendations.

The article "Impact of Dual Antiplatelet Therapy Versus Monotherapy in Acute Stroke Management: A Systematic Review" was retracted in 2025. Reasons: unreliable results or conclusions; concerns about the authorship.

Results

Study Selection Process

The study selection process, illustrated in Figure 1, followed PRISMA guidelines to ensure a rigorous and transparent approach. A total of 466 records were identified from three major databases: PubMed (n = 203), MEDLINE (n = 182), and EMBASE (n = 81). After removing 59 duplicate records, 407 records were screened based on titles and abstracts, resulting in the exclusion of 211 studies. Subsequently, 196 reports were sought for retrieval, of which 88 could not be retrieved. A thorough eligibility assessment of 108 reports was conducted, leading to the exclusion of 102 studies due to being observational or not peer-reviewed (n = 49), insufficient statistical data (n = 28), or unrelated stroke subtypes or conditions (n = 25). Ultimately, six studies met the inclusion criteria and were incorporated into the systematic review. This process highlights the comprehensive and selective approach employed to ensure high-quality evidence for the review.

**Figure 1:** The PRISMA flowchart represents the study selection process PRISMA: Preferred Reporting Items for Systematic Reviews and Meta-Analyses

Characteristics of the Selected Studies

The selected studies, summarized in Table 1, encompass a diverse range of patient populations and clinical scenarios, providing robust insights into the comparative efficacy and safety of DAPT versus monotherapy in acute ischemic stroke and TIA. These studies include large-scale trials with sample sizes ranging from 167 to 4806 patients, investigating various subgroups such as those with intracranial arterial stenosis, large artery atherosclerosis, and genetic polymorphisms. Key outcomes measured across studies include stroke recurrence, composite vascular events, functional disability, and bleeding risks. The findings consistently demonstrate the benefits of DAPT in reducing stroke recurrence and vascular events, particularly in high-risk populations, while offering insights into factors such as timing and duration of therapy initiation. These characteristics underscore the comprehensiveness and relevance of the included studies in addressing the primary objectives of this systematic review.

**Table 1:** Summary of study designs, populations, interventions, comparators, outcomes measured, statistical data, and key findings from included studies CYP2B6: Cytochrome P450 2B6; DAPT: Dual Antiplatelet Therapy; SAPT: Single Antiplatelet Therapy; TIA: Transient Ischemic Attack; HR: Hazard Ratio; CI: Confidence Interval; POINT: Platelet-Oriented Inhibition in New TIA and Minor Ischemic Stroke; mRS: Modified Rankin Scale; OR: Odds Ratio; MI: Myocardial Infarction; LAA: Large Artery Atherosclerosis; RCT: Randomized Controlled Trial

Author(s) and Year	Population	Intervention	Comparison	Outcomes Measured	Statistical Data	Key Findings
Qiu et al., 2023 [9]	2853 patients with minor stroke or transient ischemic attack in China; carriers and noncarriers of CYP2B6 polymorphisms	Aspirin plus clopidogrel	Aspirin monotherapy	Stroke recurrence within 90 days, any bleeding, 1-year follow-up outcomes	90-day stroke recurrence: 7.1% vs. 11.3% (noncarriers) and 9.7% vs. 12.2% (carriers). Adjusted HR: 0.61 (95% CI, 0.45-0.83) for noncarriers; 0.80 (95% CI, 0.54-1.18) for carriers. Any bleeding: HR 3.23 (95% CI, 0.86-12.12) for carriers.	Aspirin plus clopidogrel was effective in reducing stroke recurrence compared to aspirin alone, with a greater benefit for noncarriers. Bleeding risk was higher among carriers. No significant efficacy difference between carriers and noncarriers.
Balali et al., 2024 [10]	2559 patients with minor ischemic stroke enrolled in the POINT trial, stratified by time-to-treatment	Aspirin plus clopidogrel (DAPT)	Aspirin monotherapy	Disability at 90 days (mRS > 1) and major hemorrhage, stratified by time-to-treatment initiation	Disability rate: <6.7 h: 5.1% vs. 8.6% (OR 0.57, 95% CI: 0.33-0.99); 6.7–10.0 h: 7.5% vs. 9.9% (OR 0.74, 95% CI: 0.45-1.19); >10.0 h: 8.6% vs. 10.6% (OR 0.80, 95% CI: 0.50-1.26). Major hemorrhage: no significant difference.	Earlier initiation of DAPT (<6.7 h) was associated with a significant reduction in disability at 90 days compared to aspirin monotherapy, though no significant difference was observed in major hemorrhage rates.
Uchiyama et al., 2021 [11]	547 high-risk Japanese patients with ischemic stroke and ≥50% intracranial arterial stenosis	DAPT with cilostazol and clopidogrel or aspirin	SAPT with clopidogrel or aspirin	Recurrent ischemic stroke, composite vascular events (stroke, MI, vascular death), severe bleeding risk	Recurrent stroke: HR 0.47 (95% CI, 0.23-0.95); composite events: HR 0.48 (95% CI, 0.26-0.91); severe bleeding: HR 0.72 (95% CI, 0.12-4.30).	DAPT with cilostazol significantly reduced recurrent stroke and vascular events compared to SAPT, with no significant increase in severe or life-threatening bleeding risk in patients with intracranial arterial stenosis.
Kim et al., 2023 [12]	4806 patients with large artery atherosclerotic (LAA) stroke subtype recruited from multiple centers	DAPT (aspirin and clopidogrel) for 12 months	DAPT for 3 months, followed by monotherapy for 9 months	Composite vascular events (stroke, MI, all-cause mortality), stroke subtypes (ischemic/hemorrhagic), major bleeding	Targeting a 22% relative risk reduction with 80% power and a two-sided alpha of 0.05. Study outcomes include composite events and bleeding risk over 1 year.	Longer DAPT duration is hypothesized to reduce recurrent vascular events compared to shorter DAPT duration. The study aims to provide clarity on optimal therapy duration for LAA stroke patients. Outcome data pending trial completion.
Toyoda et al., 2022 [13]	1879 patients with high-risk non-cardioembolic ischemic stroke, stratified by timing of treatment initiation	DAPT with cilostazol and aspirin or clopidogrel	Monotherapy with aspirin or clopidogrel	Recurrence of ischemic stroke; severe or life-threatening bleeding	Stroke recurrence rates: 15-28 days group: 1.5% vs. 4.9% (HR 0.34, 95% CI 0.12-0.95); 29-180 days group: 1.9% vs. 4.4% (HR 0.27, 95% CI 0.12-0.63). Bleeding risk: HR 0.22–1.07 across groups, no significant increase.	DAPT initiated 15-180 days post-stroke was more effective than monotherapy in reducing stroke recurrence without increasing severe bleeding risk. Early DAPT initiation (8-14 days) showed no added benefit over monotherapy.
Bulwa et al., 2020 [14]	167 patients with minor ischemic stroke and ipsilateral nonstenotic carotid disease (1%-49% stenosis) compared to 833 patients without carotid disease	DAPT with aspirin and clopidogrel	Aspirin monotherapy	Recurrent ischemic stroke within 14 days, safety outcomes	Recurrent stroke in carotid disease patients: 5.4% recurrence. HR for DAPT vs. monotherapy: 0.50 (95% CI, 0.18-1.40; P=0.19). No significant safety difference noted.	Patients with ipsilateral nonstenotic carotid disease were at higher risk of early stroke recurrence. DAPT showed a numerical reduction in recurrence compared to monotherapy but was not statistically significant. Further research is needed.

Quality Assessment

The quality assessment of the included studies, as summarized in Table 2, was conducted using the Risk of Bias (RoB 2) tool (The Cochrane Collaboration, London, UK) to ensure reliability and validity. Most studies, including those by Qiu et al. [9], Balali et al. [10], and Uchiyama et al. [11], were assessed as having a low risk of bias, with robust randomization, adequate blinding, and clearly defined outcome measures, resulting in a high overall quality rating. However, studies such as Toyoda et al. [13] and Bulwa et al. [14], which involved post hoc or exploratory analyses, demonstrated moderate risks of bias due to potential selection bias, small sample sizes, or lack of predefined outcomes. Despite these limitations, the overall quality of evidence supports the reliability of the findings, with high-quality studies forming the foundation for the review’s conclusions.

The article "Impact of Dual Antiplatelet Therapy Versus Monotherapy in Acute Stroke Management: A Systematic Review" was retracted in 2025. Reasons: unreliable results or conclusions; concerns about the authorship.

**Table 2:** Evaluation of study quality using the Risk of Bias (RoB 2) tool, including study design, assessment results, and overall quality ratings of studies analyzing the efficacy and safety of dual antiplatelet therapy (DAPT) as compared to monotherapy

Author(s) and Year	Study Design	Quality Assessment Tool Used	Assessment Results	Overall Quality
Qiu et al., 2023 [9]	Randomized Controlled Trial	Risk of Bias (RoB 2)	Low risk of bias; randomization and blinding were adequate. Outcome measures were clearly defined.	High
Balali et al., 2024 [10]	Randomized Controlled Trial	Risk of Bias (RoB 2)	Low risk of bias; well-defined randomization and time stratification. Adequate handling of missing data.	High
Uchiyama et al., 2021 [11]	Randomized Controlled Trial	Risk of Bias (RoB 2)	Low risk of bias; appropriate randomization and blinding. Outcomes were predefined and consistently reported.	High
Kim et al., 2023 [12]	Prospective Randomized Controlled Trial	Risk of Bias (RoB 2)	Low risk of bias; registry-based design with clear endpoints and adequate follow-up.	High
Toyoda et al., 2022 [13]	Post Hoc Analysis of RCT	Risk of Bias (RoB 2)	Moderate risk of bias; post hoc design may introduce selection bias. Statistical analysis was robust.	Moderate
Bulwa et al., 2020 [14]	Exploratory Analysis of RCT	Risk of Bias (RoB 2)	Moderate risk of bias; exploratory nature and small sample size limit generalizability. Outcomes were not predefined.	Moderate

Discussion

The primary objective of this systematic review was to evaluate the comparative effectiveness and safety of dual antiplatelet therapy (DAPT) versus monotherapy in the management of acute ischemic stroke and TIA. The findings consistently demonstrated that DAPT provided superior outcomes in reducing stroke recurrence across various patient populations. For instance, Qiu et al. reported a significant reduction in 90-day stroke recurrence with aspirin plus clopidogrel compared to aspirin monotherapy among noncarriers of CYP2B6 polymorphisms (7.1% vs. 11.3%; HR 0.61, 95% CI: 0.45-0.83) [9]. However, the benefit was less pronounced in carriers (9.7% vs. 12.2%; HR 0.80, 95% CI: 0.54-1.18), indicating a potential genetic influence on treatment efficacy. Similarly, Balali et al. analyzed data from the POINT trial and found that earlier DAPT initiation (<6.7 hours post-stroke) significantly reduced disability at 90 days (5.1% vs. 8.6%; OR 0.57, 95% CI: 0.33-0.99) compared to aspirin monotherapy [10]. However, later initiation (6.7-10.0 hours and >10.0 hours) showed diminishing effects, highlighting the critical importance of timing in maximizing DAPT efficacy.

The article "Impact of Dual Antiplatelet Therapy Versus Monotherapy in Acute Stroke Management: A Systematic Review" was retracted in 2025. Reasons: unreliable results or conclusions; concerns about the authorship.

Further statistical analysis from other studies reinforced the benefits of DAPT in specific high-risk populations. Uchiyama et al. reported a marked reduction in recurrent stroke risk among patients with intracranial arterial stenosis treated with DAPT compared to single antiplatelet therapy (HR 0.47, 95% CI: 0.23-0.95), with no significant increase in severe bleeding risk (HR 0.72, 95% CI: 0.12-4.30) [11]. Similarly, Toyoda et al. observed that initiating DAPT 15-180 days post-stroke resulted in lower stroke recurrence rates compared to monotherapy, particularly in the 29-180 days group (1.9% vs. 4.4%; HR 0.27, 95% CI: 0.12-0.63). In contrast, early initiation (8-14 days) did not show additional benefit (HR 1.02, 95% CI: 0.51-2.04) [13]. These findings, combined with data from Kim et al. [12], which hypothesized a 22% relative risk reduction with longer DAPT duration, emphasize the nuanced role of DAPT in optimizing stroke outcomes. Collectively, the statistical data provide robust evidence supporting the efficacy of DAPT while also highlighting areas where timing, duration, and patient-specific factors significantly influence treatment outcomes.

The findings of this systematic review align with previous research demonstrating the efficacy of DAPT over monotherapy in reducing recurrent vascular events in acute ischemic stroke and TIA patients [15,16]. For instance, studies included in this review, such as Qiu et al. [9] and Uchiyama et al. [11], reported hazard ratios of 0.61 and 0.47, respectively, indicating a significant reduction in stroke recurrence with DAPT compared to monotherapy. These results are consistent with earlier meta-analyses, such as Geeganage et al. [15], which observed a risk ratio of 0.69 (95% CI: 0.60-0.80, P<0.001) favoring DAPT, and Yang et al. (2018), which reported a similar reduction in recurrent stroke risk (RR 0.69, 95% CI: 0.61-0.78, P<0.001).

However, discrepancies exist regarding bleeding risks associated with DAPT. While studies in this review, such as Balali et al. [10] and Toyoda et al. [13], found no significant increase in major hemorrhage rates, some studies highlighted an elevated bleeding risk [17]. These differences may stem from variations in study populations, treatment durations, or definitions of bleeding events. Overall, the current review supports DAPT as a superior therapeutic approach for recurrent stroke prevention, with the caveat of closely monitoring bleeding risks and tailoring treatment to individual patient profiles.

The evidence included in this systematic review is strengthened by robust methodologies, such as the use of randomized controlled trials (RCTs) across diverse populations, which ensure high-quality and reliable data. Many studies, including Kim et al. [12] and Qiu et al. [9], featured large sample sizes, enabling meaningful statistical analysis and generalizability. Additionally, the review offers novel insights, such as the timing-dependent efficacy of DAPT, as highlighted in Balali et al. [10], and the influence of genetic polymorphisms on treatment outcomes, as reported by Qiu et al. [9]. However, the findings are not without limitations. Certain studies, such as Bulwa et al. [14], involved smaller sample sizes and exploratory designs, which may limit generalizability. Furthermore, the review applied language and time filters, focusing only on English-language studies published in the last five years, which may introduce selection bias or exclude relevant older studies. Heterogeneity in patient populations, treatment durations, and outcome measures also presents challenges in drawing uniform conclusions. Despite these limitations, the review provides valuable, evidence-based insights into the comparative efficacy and safety of DAPT versus monotherapy in acute stroke management.

The article "Impact of Dual Antiplatelet Therapy Versus Monotherapy in Acute Stroke Management: A Systematic Review" was retracted in 2025. Reasons: unreliable results or conclusions; concerns about the authorship.

The findings of this systematic review hold significant clinical and practical implications, offering critical insights into optimizing treatment strategies for acute ischemic stroke and TIA management. By demonstrating the superiority of DAPT over monotherapy in reducing stroke recurrence and disability, particularly in high-risk subgroups, this review provides robust evidence to inform treatment guidelines [18,19]. Notably, the timing of therapy initiation emerged as a key factor, with early DAPT (within 6.7 hours) showing significant reductions in disability, as highlighted by Balali et al. [10,20]. Furthermore, the influence of genetic polymorphisms, as reported by Qiu et al. [9], underscores the potential for personalized medicine approaches to enhance therapeutic efficacy while minimizing risks. The novelty of this work lies in synthesizing these nuanced findings across diverse populations, offering tailored insights for patient management [21,22]. This review not only addresses gaps in the literature but also provides a foundation for refining treatment protocols, improving outcomes, and advancing the precision of stroke care.

This systematic review identifies critical gaps in the current evidence, highlighting several avenues for future research. One notable area is the need for large-scale trials to clarify the optimal duration of DAPT for different stroke subtypes, particularly in high-risk populations such as those with large artery atherosclerosis or intracranial arterial stenosis [23]. Additionally, the role of genetic polymorphisms warrants further exploration to determine how personalized medicine can optimize DAPT efficacy while minimizing bleeding risks [24]. Questions regarding the long-term safety profile of DAPT, especially concerning the balance between stroke prevention and bleeding complications, remain unresolved. Future studies should also evaluate the effectiveness of DAPT in underserved populations and non-English-speaking cohorts to address potential biases in the existing literature. Lastly, real-world evidence studies focusing on the implementation of DAPT in clinical practice could bridge the gap between trial findings and everyday patient care, offering more practical insights into its broader applicability.

The article "Impact of Dual Antiplatelet Therapy Versus Monotherapy in Acute Stroke Management: A Systematic Review" was retracted in 2025. Reasons: unreliable results or conclusions; concerns about the authorship.

## Conclusions

This systematic review highlights the efficacy of DAPT over monotherapy in reducing stroke recurrence and improving functional outcomes in patients with acute ischemic stroke or TIA, particularly in high-risk subgroups. The findings emphasize the importance of timing, with early initiation of DAPT (e.g., within 24-48 hours of symptom onset) and a short duration of therapy (typically 21-90 days) shown to maximize benefits while minimizing bleeding risks. Patient-specific factors, such as genetic polymorphisms, further influence treatment efficacy, underscoring the need for individualized approaches. While the review provides valuable guidance for refining clinical practice and treatment guidelines, it also identifies gaps in evidence such as the need for real-world studies and long-term safety evaluations. By offering a balanced interpretation grounded in robust methodologies and diverse patient populations, this review reinforces the significance of personalized, evidence-based approaches in stroke management without overstating the current evidence base.
